RETRACTED

# *Pseudomonas aeruginosa*–induced nociceptor activation increases susceptibility to infection

**DOI:** 10.1371/journal.ppat.1009557

**Published:** 2021-05-06

**Authors:** Tiffany Lin, Daisy Quellier, Jeffrey Lamb, Tiphaine Voisin, Pankaj Baral, Felix Bock, Alfrun Schönberg, Rossen Mirchev, Gerald Pier, Isaac Chiu, Mihaela Gadjeva

**Affiliations:** 1 Department of Medicine, Division of Infectious Diseases, Brigham and Women’s Hospital, Harvard Medical School, Boston, Massachusetts, United States of America; 2 Department of Immunology, Harvard Medical School, Boston, Massachusetts, United States of America; 3 Department of Ophthalmology, University Hospital of Cologne, Cologne, Germany; 4 Department of Biological Chemistry and Molecular Pharmacology, Harvard Medical School, Boston, Massachusetts, United States of America; University of Toronto, CANADA

## Abstract

We report a rapid reduction in blink reflexes during *in vivo* ocular *Pseudomonas aeruginosa* infection, which is commonly attributed and indicative of functional neuronal damage. Sensory neurons derived *in vitro* from trigeminal ganglia (TG) were able to directly respond to *P*. *aeruginosa* but reacted significantly less to strains of *P*. *aeruginosa* that lacked virulence factors such as pili, flagella, or a type III secretion system. These observations led us to explore the impact of neurons on the host’s susceptibility to *P*. *aeruginosa* keratitis. Mice were treated with Resiniferatoxin (RTX), a potent activator of Transient Receptor Potential Vanilloid 1 (TRPV1) channels, which significantly ablated corneal sensory neurons, exhibited delayed disease progression that was exemplified with decreased bacterial corneal burdens and altered neutrophil trafficking. Sensitization to disease was due to the increased frequencies of CGRP-induced ICAM-1^+^ neutrophils in the infected corneas and reduced neutrophil bactericidal activities. These data showed that sensory neurons regulate corneal neutrophil responses in a tissue-specific matter affecting disease progression during *P*. *aeruginosa* keratitis. Hence, therapeutic modalities that control nociception could beneficially impact anti-infective therapy.

## Author summary

Many of the molecular mechanisms behind bacterial keratitis induced nociception activation and specifically, how pathogen-sensing sensory neurons impact the outcome of infection have yet to be discovered, Elucidating the molecular and cellular mechanisms of nociceptor activation during bacterial keratitis can have a profound impact on treatment approaches. In this study, we established that *P*. *aeruginosa* can directly induce calcium influx in neurons and this induction is dependent on several virulence factors. Further, we demonstrated that Resiniferatoxin (RTX), a toxin that overactivates TRPV1 channels leading to chemical ablation of neurons, induces significant loss of sensory neurons in the cornea and this improves temporarily local innate responses to *P*. *aeruginosa*.

RETRACTED

## Introduction

*Pseudomonas aeruginosa* keratitis is known to cause disease with an acute onset [1–4]. If not treated appropriately and in a timely manner, this bacterial infection can lead to decreased visual acuity and even blindness. This is due to severe opacification of the cornea or ulceration, indicative of massive tissue destruction that is known to be caused by multiple factors including the inflammatory response of host, the activity of bacterial toxins, and the toxicity from antibiotic treatment. Corneal sensitivity is altered after bacterial keratitis suggestive of functional changes in neuronal activation [5]. Yet, in contrast to studies in viral keratitis, particularly in Herpes Simplex Virus and Herpes Zoster Virus infections [6–9], not much is known about the impact of nociception during bacterial keratitis. Thus, a comprehensive understanding of the impact of nociceptor activation during bacterial keratitis is crucial for developing improved therapeutic approaches.

The cornea is densely innervated with approximately 7,000 sensory neurons per square millimeter, making this tissue 300 to 600 times more sensitive to sensory stimuli than skin [5] [10–13]. The abundance of nerve terminals in this avascular environment suggests that the cornea is a unique organ with specific morphological and functional properties involved in nociception [14]. About 70% of corneal neurons are polymodal and respond to noxious stimuli such as pressure, temperature, and toxins [15] [12, 16]. The sensory neurons in the eye almost exclusively originate from the ophthalmic division of the trigeminal ganglion (cranial nerve V), which branches into nerve fibers that enter the cornea at the level of the sclera, subconjunctival and episcleral tissue, penetrating radially into the stromal substantia propria around the corneal circumference. These neurons form dense bundles that terminate into nerve endings within the corneal epithelium [17]. Corneal nerves maintain direct physical contact with corneal epithelial cells, stromal cells, and immune cells such as dendritic cells (DC) and macrophages in a tight cell-to-cell communication that is stimulated by the absence of neuronal myelination [18, 19].

The unmyelinated C-fibers of the cornea contain either peptidergic or non-peptidergic effectors [20, 21]. Once stimulated, the peptidergic sensory nerve terminals release neuropeptides including Substance P (SP), Calcitonin Gene-Related Peptide (CGRP), Neurokinin A, and neurotrophins, as well as growth factors that have been found to regulate epithelial growth and regeneration [17, 22]. In rodents, the peptidergic neurons contain 10–20% SP and 40–60% CGRP [17, 23]. The neuropeptides impact the immune/inflammatory response to corneal infection, suggesting a relationship between nociception and corneal immunity that is distinct from other sites of the body. To date, with the exception of the work on vasoactive intestinal peptide (VIP) and SP, limited number of studies have examined neuro-immune responses and the potential role of neuropeptides in regulating innate immunity to bacterial ocular infections [6, 24–28].

RETRACTED

Emerging evidence suggests that pathogens can directly activate nociceptors and elicit pain using a suite of novel and intriguing mechanisms. For example, *Staphylococcus aureus* induces pain through two mechanisms. The first involves secretion of pore-forming toxins including α-hemolysin, that causes pain by directly forming pores in dorsal root ganglia (DRG) nociceptor neurons, thus permitting cation influx and action potential generation [29, 30]. The second involves bacterial N-formylated peptides (FP) that are sensed by FPR1^+^ nociceptor neurons [30]. LPS from Gram-negative bacteria has also been found to induce nociceptor activation by neuronal TLR4 mediated sensitization of TRPV1 channels, or directly through LPS-mediated gating of TRPA1 ion channels [31, 32]. These effects are dependent on the lipid A structure, implying that distinct Gram-negative pathogens with different lipid A structures will activate different nociceptors. Aβ-fiber sensory neurons also express TLR5, allowing them to respond to bacterial flagellins [33]. Injection of bacterial flagellin together with the charged lidocaine derivative QX-314 produced significant pain blockade in models of pain emanating from chemotherapy, nerve injury, and diabetic neuropathy, providing an approach for targeted silencing of Aβ-fibers [33]. Cumulatively, these studies contribute to the mounting evidence that bacterial factors can be directly sensed by nociceptors. Except for a single study, the majority of the above-described findings were made in dorsal root ganglia (DRG) derived nociceptors, and therefore, further studies are needed to determine whether mechanisms of trigeminal ganglia (TG) derived nociceptors are comparable to DRG neurons and to understand how corneal innervation impacts host response to microbial infection [14].

Our working hypothesis was that corneal nociceptors can sense a bacterial presence, which will induce neuronal activation, the release of neuropeptides, and affect the nature of immune responses. We found that *P*. *aeruginosa* induced TG neuronal activation and release of neuropeptides which impacted the quality of innate immune responses to this pathogen, notably the immune phenotype of polymorphonuclear cells (PMNs), the magnitude of their response, and bacterial clearance. Furthermore, neuronal ablation through treatment with Resiniferatoxin (RTX), an ultrapotent capsaicin analog, which targets the TRPV1 channel, a marker of polymodal sensory fibers [34], caused neuropathy but facilitated bacterial clearance. These results suggest that treatment modalities for bacterial keratitis should evaluate their impact on neuronal responses and pain as there may be consequences from modulating neuronal responses in terms of the progression of the infection. In a broader sense, further investigations into the immune-neurologic axes that impact disease have the potential to find new treatment modalities, refine pain interventions during infections, and open new areas of investigation about how the host responds to infection.

RETRACTED

## Results

### *P*. *aeruginosa* infection causes neuropathy

To examine the impact of *P*. *aeruginosa* corneal infection on neuronal responses, corneas from C57BL6/N mice were gently scratched to allow for infection to occur, and blink responses and corneal neuronal morphologies examined. Sham-treated mice showed no significant alterations in the blink reflexes measured using the Cochet-Bonnet esthesiometer (Fig 1A). The blink reflexes of *P*. *aeruginosa* infected mice were significantly reduced and dropped from mean values of 6 to a threshold of 4, demonstrating functional impairment (Fig 1A, One-way ANOVA, p = 0.001). A further significant decrease in the blink reflexes was measured at 48h after infectious challenge reaching values less than 3 (Fig 1A, One-way ANOVA, p = 0.0001). There was a trend for the infected male mice to show lower blink reflexes than the infected female mice, but it did not reach significance. Photographs of infected corneas showed clear clinical signs of infection such as corneal infiltration and opacity which were absent in the sham-treated mice (Fig 1B).

**Fig 1:** Bacterial infection induces neuropathy. **A.** Corneal sensitivity was tested using Cochet-Bonnet esthesiometer. Infected male (N = 6) and female (N = 6) cohorts of C57BL6/N mice were compared to shams (N = 6). Changes in the blink reflexes were monitored over time (hours). The asterisks denote significant differences in blink reflexes (Two-way ANOVA, 24h, p = 0.0001; 28h, p = 0.0006; 48h, p = 0.0001). **B.** Eyes from C57BL6/N mice were either scratched (shams) (N = 6) or scratched and infected with 5x10^5^ CFU/eye *P*. *aeruginosa* 6294 (N = 6). Representative images of eye appearance at 24h and 48h post-infectious challenge are shown. The images were acquired using Motic SMZ140-143 stereomicroscope. **C.** Corneal tissues were harvested at 24h and 48h after challenge and corneal tissues were stained for β-tubulin. Z-stacks of corneal whole-mounts covering a depth of 40 μm were acquired with 1 μm step. The z- stacks were collapsed to 2D. The images are representative 2D projections. The top series of images are depicting central area of corneas while the bottom panels depict β-tubulin staining in peripheral corneas; scale bar, 20 μm. the appearance of six individual corneal whole mounts were compared per condition. **D.** Image quantification using Fiji. The 40 μm z-stacks were collapsed to 2D and areas of β-tubulin staining were calculated per slide. Data are presented with bar plots where each symbol represents the value of an individual animal. One-way ANOVA, overall p = 0.001. P values for the individual comparisons are shown on the plot. Asterisks indicate significant differences. Data demonstrate that infection changes corneal pain sensation and reduces densities of the neuronal network in central and peripheral corneas.

RETRACTED

Consistent with alterations in the blink reflexes, the β3-tubulin-specific neuronal staining of infected corneal whole mounts showed a quick collapse of the sub-basal nerve plexus in central and peripheral corneas within the first 24h of infection (Fig 1C). In contrast, in sham-treated mice the neuronal fiber densities of the sub-basal nerve plexus changed significantly less (Fig 1C, One-way ANOVA, p = 0.01), and importantly, the reductions were recovered quickly (Fig 1D). At 48 h post-scratch, the shams showed characteristic β3-tubulin staining in central corneas and regrowth of neuronal fibers in the periphery (Fig 1C and 1D), which is consistent with previous observations that corneal healing is fast in conditions of sterile wounding [35]. In contrast to the shams, the sub-basal nerve plexus of the infected mice was almost completely destroyed with changes now affecting the stromal neuronal fiber densities. The neuropathy in the infected mice was present in both, male and female infected mice. Cumulatively, our data documented that infection-induced functional neuropathy was associated with an early reduction in blink reflexes and loss of β3-tubulin-specific staining in the central and peripheral corneas.

### *P*. *aeruginosa* activates TG neurons in pili, flagella, and Type III secretion system-dependent manner

The current understanding of neuronal activation subsequent to infectious challenge suggests that it is an indirect consequence of infection-induced inflammatory responses leading to epithelial tissue destruction by secreted factors. We evaluated whether neuronal activation occurred in direct response to bacterial factors. As TG neurons innervate the cornea, we evaluated the effects of bacteria on these neurons by imaging and quantifying the intracellular calcium levels. When exposed to *P*. *aeruginosa* strain 6294, TG derived sensory neurons responded with measurable and significant Ca^2+^ fluxes (Fig 2A and 2B). Overall, about 50% of the neurons responded to bacteria with Ca^2+^ fluxes, demonstrating selective activation. There was also significant overlap between *P*. *aeruginosa*–induced neuronal activation and capsaicin-triggered responses (Fig 2C). About 50% of the capsaicin-activated neurons also responded to *P*. *aeruginosa* (Fig 2C). These findings suggest that TRPV1-expressing (capsaicin-responsive) neurons can fire upon *P*. *aeruginosa* exposure. This further suggests that the *P*. *aeruginosa* induced nociception can be prompted by a direct contact between a neuron and bacteria.

RETRACTED

**Fig 2:** *P*. *aeruginosa* 6294 activates trigeminal neurons. Trigeminal ganglia were harvested from C57BL67/N mice; cultured neuronal cells (see text) were exposed to live *P*. *aeruginosa* 6294 (MOI 10), capsaicin, and potassium chloride (KCl). Calcium influx into the neuronal cells was imaged in real-time using Fura-2 AM dye. Capsaicin activated TRPV1 firing; KCl activated all neurons. **A.** Representative confocal images of neuronal cells responding to stimuli acquired at 40x magnification; scale bar, 50μm. Neurons were imaged for 30 minutes. The appearance of green or red neuronal cells (arrows) indicates increase of intracellular Ca^2+^ levels proportionally to the degree of activation in real-time (color bar: fluorescence intensity, arb. units). **B.** Representative time course of calcium traces in activated neurons in one of two independent experiments. Time course is followed measuring normalized fluorescence intensity 340/360 ratio. Black arrows indicate the time point of application of 6294, capsaicin, and KCl. **C.** Bar graph depicts the total number of responding neurons per field of view at 10x magnification. The first bar indicates percent of neurons responding to bacteria; values are mean +/-SD. The second bar depicts the number of neurons responding to *P*. *aeruginosa* that also respond to capsaicin stimulation. Cumulatively, data show that similar numbers of TG neurons respond to capsaicin and *P*. *aeruginosa*. **D.** Representative whole-mount ocular image shows the proximity of bacteria and neuronal fibers. Mice expressing a red fluorescent protein under the NaV 1.8 promoter (Nav 1.8^cre^/TdTomato, red) were infected with 5x10^5^ CFU/eye GFP-expressing *P*. *aeruginosa* 6294 (Green). The scale bar is 20μm. Cumulatively, these data demonstrate that *P*. *aeruginosa* induces Ca^2+^ influxes in neurons, reflective of activation.

RETRACTED

The sodium channel NaV1.8 is a marker of the majority of nociceptive sensory neurons, which mediate cold, mechanical, and inflammatory pain [36]. Confocal microscopy of corneas from NaV1.8 ^cre^/TdTomato mice which express the red fluorescent protein TdTomato under the NaV1.8 Cre promoter visualized the proximity of *P*. *aeruginosa* 6294 expressing GFP with sensory neurons expressing the NaV1.8 sodium channel (Fig 2D).

To determine which *P*. *aeruginosa* factors may be associated with this neuronal response, infections with *P*. *aeruginosa* strain PAK (wild-type), pili knockout strain PAK Δ*pilA*, flagella knockout strain PAK Δ*fliC* and type III secretion system (T3SS) knockout PAK Δ*exsA* were evaluated. While TG neurons responded strongly to wild-type strain PAK, the neurons had a minimal or no response to PAK Δ*pilA*, Δ*fliC*, and Δ*exsA* mutants, indicating that Ca^2+^-flux-based responses to *P*. *aeruginosa* were dependent on virulence factors associated with mobility and T3SS-induced cellular activation (Fig 3). We presume that for T3SS activation and delivery of the intracellular effectors mobility is essential to bring the bacterial cells in close proximity to neurons.

**Fig 3:** *P*. *aeruginosa* virulence factors pili, flagella, and T3SS trigger neuronal activation. **A.** Representative confocal images of neuronal activation by PAK (first row), PAK Δ*pilA* (second row), PAK Δ*fliC (*third row*)*, and PAK Δ*exsA (*forth raw*)* strains of *P*. *aeruginosa*. Images were acquired at 10x magnification. Scale bar, 100 μm. Trigeminal ganglia were harvested from C57BL6/N mice and neuronal cultures were grown *in vitro*. Cultures were activated by exposure to live *P*. *aeruginosa* PAK or mutant strains, capsaicin, and potassium chloride (KCl). Neuronal cell activation was imaged for 30 min. Appearances of green or red neuronal cells (arrows) are indicative of activation. Capsaicin activates TRPV1-carrying neurons. KCl activates all live neurons. The arrows point to neuronal cells responding to stimulation. Note the appearance of green cells upon *P*. *aeruginosa* PAK stimulation (second image, first raw); the color changes to red upon capsaicin stimulation, illustrating the response of capsaicin-sensitive TRPV-1^+^ nociceptors. The transition from green to red indicates increase in the strength of Ca^2+^ fluxes activation (see also caption under Fig 2). Expectedly, capsaicin application after *P*. *aeruginosa* stimulation elevates Ca^2+^ fluxes. **B.** Percent of neurons responding to different strains of *P*. *aeruginosa*. Responding cells were characterized as neurons that displayed a signal 25% higher than the baseline. Significantly fewer neurons responded to *exsA*, *pilA*, and *fliC* mutants when compared to neurons responding to PAK WT (Overall one-way ANOVA p<0.05, p-values indicate comparisons to PAK WT exposure (Cntrl) using Dunnett’s pairwise comparison test). **C.** Venn diagrams of numbers of *P*. *aeruginosa*–induced responding neurons and capsaicin-responding neurons per analysis. The overlap between capsaicin-responding neurons and *P*. *aeruginosa*-responding neurons indicates that TRPV1^+^ neurons can be activated after *P*. *aeruginosa* stimulation. Data show that virulence factors governing bacterial motility or T3SS promote neuronal activation.

RETRACTED

### RTX treatment ameliorates disease and changes neutrophil recruitment and functionality in the cornea

Resiniferatoxin (RTX) is an ultrapotent capsaicin analog that causes chemical denervation of TRPV1^+^ neurons [37, 38]. We reported previously that administration of RTX to 4-week-old mice resulted in destruction of TRPV1^+^ neurons and lasting systemic denervation in the skin and gut [39, 40]. We used this model system to examine the impact of RTX-responding neurons on immunity to *P*. *aeruginosa*–induced keratitis.

Analysis of ocular blink reflexes in RTX-treated mice revealed a mild but significant reduction in reflexes at 1-week post-RTX treatment, followed by complete recovery (Fig 4C, Two-way ANOVA, asterisk, p = 0.003), exemplifying lack of changes in mechanosensitivity. While corneal blink reflexes were not significantly affected, the RTX treatment led to a significant reduction in eye wipe reflexes upon stimulation of TRPV1^+^ nociceptors with capsaicin (S1 Fig, Student’s *t*-test, p = 0.0125). The application of capsaicin onto corneas of vehicle-treated mice stimulated eye wiping behavior, which was significantly reduced in the RTX-treated mice, consistent with the expected reductions of TRPV1^+^ neurons that respond to capsaicin. Cumulatively, data showed that selective ablation of RTX-responsive neurons does not trigger functional side effects associated with lasting reductions in blink reflexes (Fig 4).

**Fig 4:** RTX treatment reduces bacterial burden in the infected eyes. **A.** Schematic representation of the experimental approach. Subcutaneous inoculation of RTX was given to four-week-old mice. The mice were treated for 3 consecutive days, with incrementing dosages; day one: 30 μg/kg; day two: 70 μg/kg; day three: 100 μg/kg. Mice were rested and infected at 6 weeks of age with 5x10^5^ CFU/ml of *P*. *aeruginosa* 6294. Ocular tissues were harvested for analysis. **B.** Representative images of sham (left) and infected (right) eyes at 24h post-challenge. Data are representative from three independent experiments with N = 6 mice per treatment per experiment. **C.** Corneal sensitivity was captured by measuring the blinking thresholds of mice longitudinally, commencing with RTX treatment and ending with infection. The RTX treatment caused a mild, but significant decrease of blinking reflexes (asterisk, p = 0.003, Two-way ANOVA) that was observed only a week post-treatment, followed by complete recovery. The blinking threshold significantly declined in infected mice under both treatments. Data are representative from three independent experiments with N = 6 mice per treatment per experiment. **D.** Representative images of stained for β-tubulin shams and infected corneal whole mounts from RTX- and vehicle-treated mice, scale bar = 20 μm. The z-stack covers 40 μm from corneal epithelium to stroma with 1 μm interval and is shown as 2D projection. The images were analyzed using custom script in Fiji to quantify stained areas per image. Six whole-mounts per group per treatment were analyzed and values plotted (right panel; p-values by One-way ANOVA; ns, not significant). The quantification of β-tubulin-stained areas shows decrease of β-tubulin in cornea periphery upon RTX treatment and with infection. **E.** Mouse scratch-injured corneas were infected with 5x10^5^ CFU/ml of *P*. *aeruginosa* 6294 and corneal and conjunctival tissues were harvested at 24h post-challenge. Bacterial burdens were determined by plate counts **(**Student’s *t*-test, p = 0.0001). Corneal pathology was depicted by box and whiskers plots showing 25% and 75% ranges (Mann-Whitney comparison, p = 0.01). Data are representative from three independent experiments, each containing cohorts with N = 6 mice per treatment per experiment. Cumulatively, data show that the reduction in neuronal fibers abundance consequent to RTX treatment did not cause sustained alterations in blink reflexes. Significant changes in pain sensation were observed only consequent to infection irrespective of RTX treatment. RTX treatment resulted in decreased *P*. *aeruginosa* burden in the infected corneas.

RETRACTED

Next, we assessed the impact of RTX injection on potential cellular infiltration in the eyes of resting mice. The immunohistochemical analysis of ocular tissues did not show major changes in numbers of Ly6G^+^ myeloid cells, CD3^+^, CD8^+^ cells, or MHCII^+^ antigen-presenting cells in unchallenged mice (S2, S3 and S4 Figs). Cumulatively, these data revealed that the RTX-treatment did not induce overt inflammatory responses at baseline despite the detectable abrogation of RTX-responsive nociceptors.

Scratched RTX-treated mice displayed expected reductions in sub-basal nerve plexus β-tubulin^+^ staining when compared to vehicle-treated shams (Fig 4D, One-way ANOVA, p<0.0006) (S1 and S2 Videos). When infected, the RTX injected and vehicle-treated mice exhibited further reductions in neuronal fibers occurring 24h post-bacterial-challenge (Fig 4D, S3 and S4 Videos). The infected RTX- and vehicle-treated mice showed similar decrease in blink reflexes (Fig 4C). Interestingly, the infected corneas from the RTX-treated mice had a 1-log reduction in bacterial burden at 24 hours of infection (Fig 4E and 4B). These data point to alterations of the response to bacterial challenge in the absence of RTX-responsive neurons.

Myeloid cell trafficking and functionality are major determinants of immune protection. At 24h post-infectious challenge, we observed differences in the total numbers, frequencies, and characteristics of infiltrating myeloid cells in the infected corneas. Corneal cellularity was significantly elevated in the infected RTX-treated mice as absolute cell counts of CD45^+^ cells and myeloid CD11b^+^Ly6G^+^ cells were increased when compared to the infected vehicle-treated mice, consistent with activation of the inhibitory effects of nociceptors on cellular infiltration (Fig 5B, Student’s *t*-test, p = 0.0001). Infected RTX-treated mice showed increased frequencies of CD45^+^ cells, CD11b^+^Ly6G^-^ cells, and CD11b^+^Ly6G^+^ myeloid populations (Fig 5B, Student’s *t*-test, p = 0.001, p = 0.001, and p = 0.002). Two different populations of CD11b^+^Ly6G^+^ myeloid cells could be distinguished depending on levels of expression of ICAM-1 expression: Ly6G^+^CD11b^+^ ICAM-1^-^ and Ly6G^+^CD11b^+^ ICAM-1^+^ cells. The Ly6G^+^ CD11b^+^ ICAM-1^-^ population of neutrophils, was enriched in the infected RTX-treated mice (Fig 6A, Student’s *t*-test, p = 0.001), whereas the Ly6G^+^CD11b^+^ICAM-1^+^ population was increased in the vehicle-treated mice (Fig 6A, Student’s *t*-test, p = 0.01). ImageStream analysis of infected mice showed that the Ly6G^+^ CD11b^+^ ICAM-1^-^ and the the Ly6G^+^CD11b^+^ICAM-1^+^ populations had banded or multilobed nuclei typical for neutrophils (Fig 6B). Hence, two different populations of neutrophils are present in the infected corneas. Phagocytosed *P*. *aeruginosa* could be detected in both populations. In contrast to the infected corneas, significantly lower and almost undetectable levels of surface ICAM-1 on Ly6G^+^CD11b^+^ cells (S5 Fig) were measured in blood and bone marrow of infected mice. Cumulatively, these data illustrate tissue-specific neuronal regulation of myeloid responses during infection.

RETRACTED

**Fig 5:** Neutrophil recruitment is increased in RTX-treated corneas. **A.** Flow cytometry analysis of cellular infiltrates in infected corneas from RTX-treated and vehicle-treated mice. Panels describe the gating strategy to identify myeloid subpopulations. PMNs were defined on FSC vs SSC gate, as CD45^+^, live cells that express CD11b and Ly6G. **B.** Quantification of the absolute cell counts reflecting populations of total CD45^+^ infiltrates (first panel), Ly6G^+^CD11b^-^ (second panel) and Ly6G^+^CD11b^+^ (third panel, neutrophils). Bar graphs show mean values; symbols represent individual mouse. Data are from N = 6 infected corneas (1 per mouse) per condition representative of two independent experiments. P-values by Student’s *t*-test. Cumulatively, data show increased cellularity in the infected RTX-treated mice.

**Fig 6:** RTX treatment reduces the frequencies of CD11b^+^ Ly6G^+^ICAM-1^+^ myeloid cells in the infected corneas. **A.** Histogram plots show gating and frequencies of CD11b^+^ Ly6G^+^ICAM-1^-^ and CD11b^+^Ly6G^+^ ICAM-1^+^ cells. Data represent 6 infected corneas (1 per mouse) per condition per cohort. The experiment was repeated twice. Bar graphs show mean values; symbols represent individual mouse. P-values by Student’s *t*-test. **B.** Representative ImageStream images of CD11b^+^ Ly6G^+^ICAM-1^+^ and CD11b^+^ Ly6G^+^ ICAM-1^-^ cells. Mice were infected with 5×10^5^ CFU of GFP-expressing *P*. *aeruginosa* 6294 (Green) per cornea; tissue was harvested at 24h post-challenge for analysis. Cellular suspensions were prepared with collagenase digestion and stained for CD45, CD11b, Ly6G, ICAM-1, and DNA (Hoechst) to identify myeloid infiltrates. CD11b^+^ Ly6G^+^ cells show banded or multi-lobed nuclear morphology typical of neutrophils. **C.** Quantification of CD11b^+^ Ly6G^+^ICAM-1^+^ and CD11b^+^ Ly6G^+^ ICAM-1^-^ myeloid cells containing intracellular *P*. *aeruginosa*-GFP (p-values by one-way ANOVA). Cumulatively, data show that nociceptor presence alters myeloid phenotypes in the infected corneas, enriching for CD11b^+^ ICAM-1^+^ Ly6G^+^ myeloid cells in vehicle-treated mice when compared to RTX-treated mice.

At 48h post-infection, the RTX treatment had no effect on the bacterial burdens, disease pathology, or inflammatory responses (S6 Fig). Cumulatively, these data demonstrate that neuronal activation likely suppresses host innate immunity in the early phases of infection before irreversible loss of neuronal fibers in the central and peripheral corneas has commenced.

RETRACTED

### CGRP inhibits neutrophil responses to *P*. *aeruginosa*

CGRP is a neuropeptide expressed by TRPV1^+^ nociceptors that is released during neuronal activation and mediates neurogenic inflammation [31]. Since the majority of the TRPV1^+^ nociceptors contain endogenous CGRP [41], depletion of these neurons results in an expected decrease in tissue CGRP illustrated by reduced neuropeptide staining in the sub-basal neuronal plexus of corneal whole mounts from sham-treated mice (Fig 7A and 7B, Student’s *t*-test, p = 0.01). The activation of TRPV1^+^ neurons by agonists triggers Ca^2+^ influx leading to immediate CGRP exocytosis from neuronal dense core vesicles [42]. We found that TG neurons exposed to *P*. *aeruginosa* strain 6294 released significantly higher levels of CGRP as compared to resting neurons in culture (Fig 7C, Student’s *t-*test, p = 0.03). To determine if exposure to CGRP affects myeloid phenotypes, purified bone marrow-derived CD11b^+^Ly6G^+^ myeloid cells (neutrophils) were incubated *in vitro* with increasing concentrations of CGRP or another nociceptive neuropeptide, SP, and percentages of ICAM-1^+^ Ly6G^+^ CD11b^+^ cells were quantified by flow cytometry (Fig 7D, One-way ANOVA, overall p = 0.003). CGRP treatment led to a significant upregulation of surface ICAM-1 with about 20% more myeloid cells expressing membrane ICAM-1 (Fig 7D, One-way ANOVA, p = 0.03). In contrast, pre-treatment with SP did not result in upregulation of ICAM-1.

**Fig 7:** CGRP inhibits bactericidal activities of neutrophils. **A.** RTX treatment reduces CGRP levels in sham-treated corneas. Representative images of CGRP staining of corneal whole-mounts from RTX and vehicle-treated shams. Z-stacks were collected from cornea periphery using Zeiss LSM710 confocal microscope with a 40x objective, scale bar = 20 μm. The z-stacks were collapsed to 2D and images were analyzed using Fiji software to quantify stained areas per image. The Z-stacks comprised sub-basal nerve plexus and stromal nerves spanning a depth of 40μm. Eight whole mounts per group per treatment were analyzed (Student’s *t*-test, p = 0.01). Each value represents an individual animal. **B.** The quantification of CGRP stained areas shows a decrease of CGRP staining in the sub-basal neuronal fibers of cornea periphery of RTX sham-treated mice when compared to sham vehicles. **C.** *P*. *aeruginosa* 6294 infections significantly induced CGRP release in trigeminal ganglia (TG)-derived neuronal cultures. CGRP concentrations were measured in the supernatants by ELISA. Bars represent means of individual mice values (symbols; Student’s *t*-test, p = 0.03). Saline treatment was used as control. Data are representative of two experiments. **D.** Exposure to CGRP, but not Substance P, upregulates membrane ICAM-1 in BM-derived neutrophils exposed to *P*. *aeruginosa*. PMNs were pretreated with 100 nM, 500 nM CGRP, or 100nM Substance P for 6h, then exposed to *P*. *aeruginosa* 6294 at MOI 0.01 for 30 min. Cells were washed, Fc blocked, and stained for ICAM-1^+^, CD11b^+^, Ly6G^+^, and 7AAD. Viable, Ly6G positive cells were compared for ICAM-1 levels. Percent ICAM-1^+^ cells were plotted. Data represent mean values. The experiment was repeated twice. **E.** CGRP inhibits bactericidal function of neutrophils. Data from three independent experiments are combined; each symbol represents cells derived from an individual mouse. One-way ANOVA, Dunnett’s multiple comparison test, p = 0.02 and p = 0.03. **F.** CGRP antagonist decreases bacterial burden in the infected corneas and conjunctival tissues. C57BL/6 mice were infected with *P*. *aeruginosa* 6294 at 5x10^5^ CFU/eye. BIBN4096 (30 mg/kg) or vehicle were injected intraperitoneally one hour after the infectious challenge. Corneal and conjunctival tissues were harvested at 24h. Symbols represent individual mice. 10 mice per cohort were analyzed. Vehicle-treated mice had significantly higher bacterial presence when compared to BIBN4096-treated mice, illustrating CGRP-driven inhibition of immunity to *P*. *aeruginosa* (Student’s *t*-test, p = 0.02) (first plot). BIBN4096 treatment moderately reduced corneal pathology in the infected mice (Mann-Whitney, p = 0.003). Cumulatively, data show that *P*. *aeruginosa* induces CGRP release by neuronal cells *in vitro* and that blockade of CGRP *in vivo* partially resembles the phenotype of the infected RTX-treated mice displaying lower bacterial presence during early hours of infection. The phenotype is likely due to reduced opsonophagocytic killing in the presence of CGRP and correlates with upregulation of ICAM-1 in neutrophils.

RETRACTED

To determine whether CGRP altered bactericidal activities, increasing doses of CGRP were added to *in vitro* CD11b^+^Ly6G^+^ BM-derived cultures stimulated with *P*. *aeruginosa*. CGRP significantly reduced the killing of *P*. *aeruginosa* (Fig 7E, One-way ANOVA and Dunnett’s pairwise comparison, p = 0.02 and p = 0.03 respectively). Although this *in vitro* inhibition was moderate, additional supportive data was generated by treating *P*. *aeruginosa* 6294 challenged mice with the CGRP antagonist BIBN4096 one hour after the *in vivo* bacterial challenge (Fig 7F). An approximate two-fold lower bacterial burden was detected in the CGRP-neutralized cohort when compared to the vehicle cohort (Fig 7F, Student’s *t*-test, p = 0.02) along with a reduction in the corneal pathology score (Fig 7F, Mann-Whitney U test, p = 0.0032), indicating that inhibition of CGRP-induced signaling improves the host clearance and corneal pathology outcomes following infection with this pathogen by likely altering neutrophil functionality.

## Discussion

*P*. *aeruginosa* is an opportunistic pathogen that often infects contact lens wearers or follows ocular trauma [43, 44]. It is thought that disturbances of the ocular surface barrier sensitize to disease [45]. Indeed, exposure of intact corneas to high dose inoculum containing *P*. *aeruginosa* is not infectious, illustrating barrier-mediated protection of the eye [46–49]. It is not fully understood why injured corneas are sensitized to disease. It is possible that wounding facilitates bacterial access to neuronal fibers in the absence of healthy barrier. To this end, we show that *P*. *aeruginosa* can activate neuronal fibers directly to trigger CGRP release, thereby further inhibiting timely innate responses.

We found that the direct interaction between *P*. *aeruginosa* and sensory neurons is dependent on the role of flagella, pili, and T3SS as virulence factors. The presence of pili promoted nociceptor Ca^2+^ fluxes, suggesting that pili can serve as tissue-specific virulence factors during ocular infections. Consistently, in the eye, *P*. *aeruginosa* type IV pili deficient strains induce less disease [50], and pili facilitate corneal epithelial traversal, a critical process for establishing infection [51]. In contrast to the eye, in the lungs, pili-deficient strains show increased fitness as measured by enhanced bacterial burdens and ability to outperform piliated wild type strains for survival [52, 53]. Cumulatively, these results point to tissue-specific pili-induced responses during *P*. *aeruginosa* infection. In the eye, pili-induced nociceptor activation is associated with increased neuropeptide release. Overall, these findings provide novel insights into the mechanisms of *P*. *aeruginosa*–established infection, namely, that by activating nociceptor signaling, *P*. *aeruginosa* suppresses initial innate responses.

In the infected mice, we observed a rapid loss of neuronal fibers in the central and peripheral cornea. The infection-induced neuropathy was sustained unlike the changes observed in the sham-treated mice. The reduction in densities of the subbasal nerve plexus correlated with a reduction in blink reflexes. While we are not aware of other studies that explore the kinetics of changes occurring in neuronal network densities during *P*. *aeruginosa*–induced keratitis, corneal imaging of patients suffering from *Acanthamoeba*–induced keratitis and HSV–induced keratitis showed profound diminishment of subbasal nerve plexus occurring within days of acute disease onset [54–57]. Cumulatively, the clinical data and animal model-based data show a quick collapse of subbasal plexus during bacterial and viral infections. An important inference from these observations is the need to evaluate the role of neuronal activation, which likely precedes neuronal loss, during disease onset and examine the implications for therapy.

RETRACTED

Neuronal activation impacted the pathogenesis of *P*. *aeruginosa*–induced keratitis and altered disease progression (Fig 8). When TRPV1^+^ nociceptors were depleted through the use of RTX, the mice displayed decreased corneal bacterial burdens and delayed disease compared to vehicle-treated controls. The phenotype was specific to the cornea, while similar approaches to ablate nociceptors did not alter sensitivity to *P*. *aeruginosa*–induced pneumonia in the lungs [58]. The findings thus demonstrate that the regulation of anti-bacterial responses by neurons is occurring in an organ-specific manner. Given the significant differences in the levels of innervation of the cornea and lung tissues [59], disease outcomes likely relate to differences in both the level of nociceptor activation and the specifics. Cumulatively, our data have significant implications as they point to site-specific therapies governed by the type of innervation present in a given tissue.

**Fig 8:** Schematic model depicting the impact of neuronal regulation on *P*. *aeruginosa* induced keratitis. *P*. *aeruginosa* utilizes flagella, pili, and type III secretion systems to initiate neuronal activation. As a result, the threshold of activation of Transient Receptor Potential Cation Channel, subfamily V, member 1 (TRPV1) is reduced increasing the excitability of the peripheral terminal membrane. When a threshold of depolarization is reached, voltage-gated sodium channels (e.g., NaV1.8) are activated and an action potential is produced and is propagated along the axon. An influx of calcium through voltage-gated calcium channels (VGCC) triggers the release of neuropeptides including calcitonin-gene-related protein (CGRP), which controls myeloid responses in the corneas. CGRP inhibits myeloid infiltration to the tissues and alters myeloid phenotypes in response to infection. The ICAM-1^+^ Ly6G^+^ CD11b^+^ neutrophils have decreased ability to kill bacteria.

A downstream event that follows *P*. *aeruginosa* activation of nociceptors is the release of CGRP [29]. CGRP signaling reduced neutrophil recruitment and bactericidal activities during invasive *Streptococcal and S*. *aureus* skin infections [39, 60] which is consistent with our data that loss of RTX-targeted nociceptors correlated with elevated corneal myeloid cellularity in infected RTX-treated mice [58]. Neutrophil recruitment and activation are major determinants of host responses against *P*. *aeruginosa* infection. Our findings that nociceptor-released CGRP temporarily inhibited innate immune responses in the cornea suggest that the nociception-induced control over innate immunity may delay efficient myeloid responses in the eye sensitizing to infection.

RETRACTED

Because elevated myeloid cell infiltration in infected corneas are often associated with inflammation-induced tissue damage and worse disease pathology, it is puzzling why in the infected RTX-treated mice, despite increased cellular infiltration, there appears to be less bacterial presence and less pathology. Given that the phenotype is observed early during infection, it is likely that the temporary increase in myeloid cells offers improved initial control over the bacterial spread. The composition and functionalities of the myeloid infiltrates differed between infected RTX- and vehicle-treated mice. We detected two distinct Ly6G^+^, CD11b^+^ populations, which varied in granularity and levels of expression of the activation signaling receptor ICAM-1. Previously, ICAM-1 positive neutrophils’ presence has been reported in sepsis and was associated with elevated ROS production and NETosis, therefore associated with heightened inflammation and emanating tissue damage [61, 62]. In humans, ICAM-1 positive neutrophils tended to aggregate as ICAM-1- interactions with Mac-1 promoted neutrophil clustering [63]. Interestingly, RTX treatment reduced the frequencies of ICAM-1^+^CD11b^+^Ly6G^+^ cells in the infected corneas, exemplifying how changes in neuronal presence affect myeloid responses as the infection continues. Further, CGRP caused upregulation of ICAM-1 on neutrophils from BM and decreased bactericidal activities. Hence, our data supported the conclusion that the appearance of ICAM-1 on neutrophils is a tissue-specific response in the infected corneas that is controlled by nociceptors.

Our work prompts questioning if the current therapeutic modalities should control downstream TRPV1 signaling and target neuropeptide, such as CGRP, release in response to infection. The experiments using the CGRP antagonist BIBN4096 showed improved bacterial clearance, supporting the idea that the use of this non-peptide compound may have therapeutic implications. Of note, BIBN4096 has been approved for human use in treatment of migraine [64].

Overall, this study highlights a previously underappreciated role for pathogen-induced neuronal regulation in the cornea that critically affects innate immunity. Further studies are needed to fully understand neuro-immune crosstalk within the context of an infectious stimulus to design organ-specific treatment modalities.

RETRACTED

## Materials and methods

### Ethics statement

All animal experiments were performed following National Institutes of Health guidelines for housing and care of laboratory animals and performed in accordance with institutional regulations after protocol review and approval by the BWH Animal Care and Use Committee and were consistent with the Association for Research in Vision and Ophthalmology guidelines for studies in animals. The experiments were carried out under the approved protocol number 2018N000002.

### Mice

C57BL6/N mice were housed in an AAALAC-approved Laboratory Animal Care Facility at Brigham and Women’s Hospital and were purchased from Taconic Farms. The Nav 1.8^cre^/TdTomato (on C57BL6N background) mice were maintained at the BWH MCP animal facility. For all experiments with Nav 1.8^cre^/TdTomato mice, littermate age and gender-matched CFU controls were used. Initially, both genders were used in the experiments. When no differences in the phenotypes were detected, only female mice were evaluated. Euthanasia was done by an overdose of CO_2_, followed by a secondary mechanism of cervical dislocation.

### Bacterial strains and inoculum

Invasive *P*. *aeruginosa* strains 6294, PAK, PAK Δ*pilA*, PAK ΔexsA, PAK Δ*fliC* were used throughout these experiments. The bacterial strains were grown overnight at 37°C on BD BBL prepared plated Media (Trypticase Soy Agar (TSA) with 5% Sheep Blood, cat. B21261X, Fisher Scientific, Pittsburg, PA, USA). The bacterial suspensions were prepared in saline solution (cat. 50-843-141, USP grade, Fisher Scientific, Pittsburg, PA, USA) and used for subsequent infection experiments.

### Infection model

Infections were carried out as described previously [65]. Briefly, mice were anesthetized with intraperitoneal injections of ketamine (cat. 9950001, Henry Schein, Albany, NY, USA) and xylazine (cat. 1311139, Henry Schein, Albany, NY, USA). Three 5 mm scratches were made on the cornea with a 25G needle and an inoculum of 5 x 10^5^ cfu of *P*. *aeruginosa* in 5 μl was delivered onto the eye. Mice remained sedated for approximately 30 min. For evaluation of corneal pathology, daily scores were recorded by an observer unaware of the experimental status of the animals based on the following scoring system using a graded scale of 0 to 4 as follows: 0, eye macroscopically identical to the uninfected contra-lateral control eye; 1, faint opacity partially covering the pupil; 2, dense opacity covering the pupil; 3, dense opacity covering the entire anterior segment; and 4, perforation of the cornea, phthisis bulbi (shrinkage of the globe after inflammatory disease), or both. To determine corneal bacterial counts at 24h or 48h after infection, mice were sacrificed, the eyes were enucleated, and the corneas were dissected from the ocular surface. To quantify the level of *P*. *aeruginosa* presence, corneas were suspended in phosphate-buffered saline (PBS, cat B220, BostonBioProducts, MA, USA), 0.05% Triton X100 (cat. 2315025, SigmaAldrich, St. Louis, MO, USA), serially diluted and plated on *P*. *aeruginosa* selective MacConkey agar plates (cat. 221270, Owens & Minor, Franklin, MA, USA).

RETRACTED

### Cytokine analysis

Levels of mouse cytokines IL-1β, MPO, MIP-2, NE, KC, and IL-6 in corneal lysates were determined using Quantikine and Duoset ELISA kits according to manufacturer’s instructions (cat. MLB00C, DY3667, MM200, MELA20, MKCOOB, M6000B, R&D Systems Inc, Milford, MA, USA).

### Flow cytometry

Individual corneas were minced and digested in 5 ml of 2 mg/ml Collagenase D (cat. 11088858001, Sigma-Roche, St. Louis, MO, USA), 0.1mg/ml DNase I (cat. 79254, QIAGEN Inc, Germantown, MD 20874), 0.7 mg/ml calcium chloride in HBSS (cat. 14025134, Fisher Scientific, Pittsburgh, PA, USA), 5% FBS, 10mM HEPES (cat. 15630106, Fisher Scientific, Pittsburgh, PA, USA) for up to 1h at 37^O^ water bath with intermittent mixing. The reaction was stopped by the addition of 5 mM EDTA (cat. AAA1071336, Fisher Scientific, Pittsburgh, PA, USA); cells were spun down at 300g for 5 min at 4° C; resuspended in FACS staining buffer containing 5% BSA (cat. 12–657 Millipore/Sigma, St. Louis, MO, USA), PBS; strained through 0.7 um filters to reduce clumping and stained for analysis. The following antibodies were used: Fc block-Anti mouse CD16/32 (cat. 14-0161-86, eBiosciences/ThermoFisher Scientific, Pittsburgh, PA, USA,), anti-mouse CD11b-PE (cat. 101207, clone M1/70, BioLegend, Dedham, MA, USA), anti-mouse Ly6G-APC (cat. 127613, clone 1A8, BioLegend, Dedham, MA, USA), pacific blue anti-mouse ICAM-1 (CD54) (cat. 116115, clone YN1/1.7.4, BioLegend, Dedham, MA, USA), anti-mouse CD45 FITC (cat. 368508, clone 2D1, BioLegend, Dedham, MA, USA). Isotype controls included rat IgG1 FITC (cat. 11-4714-42 Thermo Fisher Scientific, Pittsburgh, PA, USA), rat IgG2b-PE (cat. 12-4031-82, Thermo Fisher Scientific, Pittsburgh, PA, USA), rat IgG2a-APC (cat. 554690, BD Biosciences, San Jose, CA, USA), rat IgG2b-pacific blue (cat. RTK 4530, BioLegend, Dedham, MA, USA). Cellular viability was analyzed using 7AAD (cat. 420403, BioLegend, Dedham, MA, USA) staining. Flow cytometry laser settings were established using UltraComp eBeads beads (cat. 01-3333-41, Life Technologies/Thermo Fisher Scientific, Pittsburgh, PA, USA) labeled with the above-listed antibodies per the manufacturer’s instructions. The acquisition was carried out on Cytek DxP12 flow cytometer and the analysis was carried out in FlowJo 10.6.2.

RETRACTED

### Purification of PMNs and bactericidal assays

Murine bone marrow was flushed from both hind limbs with PBS supplemented with 2% Fetal Bovine Serum and 1 mM EDTA. The cells were washed, erythrocytes in the cell pellet were lysed using the red cell lysis buffer (cat. BUF04B, Biorad, Hercules, CA, USA) according to the manufacturer’s instruction, and neutrophils were isolated using the EasySep Mouse Neutrophil Enrichment Kit (cat. 19762, StemCell, Vancouver, Canada). For mouse serum, murine cardiac blood was collected with a syringe and a 26G needle and subsequently spun down at 4.6 rpm at 15°C for 24 minutes. Neutrophils were incubated with *P*. *aeruginosa* strain 6294 at an MOI of 100:1 with 10% mouse serum in Hanks Balanced Salt Solution containing calcium and magnesium (HBSS^+/+^) (cat. SH3058802, Fisher Scientific, Hampton, NH, USA) for 90 min at 37°C on a rotator. Rat CGRP (cat. 1169, Tocris, Bristol, UK) was added to cultures immediately before 6294 at concentrations 100 nM, 500 nM, and 1 mM. Aliquots were taken at time 0 and 90 min, serially diluted and plated on MacConkey agar to determine numbers of live *P*. *aeruginosa*. The percentage of killing ability of neutrophils was calculated as in [66].

### Resiniferatoxin treatments

To chemically ablate TRPV1^+^ neurons, C57BL/6 female mice were treated with RTX (cat. R8756, Sigma-Aldrich, St. Louis, MO, USA). Four-week-old mice (with an average weight of 17 grams) were anesthetized by inhalation of isoflurane and injected subcutaneously with the following dosages over three consecutive days: 30 μg/kg, 70 μg/kg, and 100 μg/kg [31]. Control littermates were injected with vehicle solution (0.5% EtOH, 1% EtOH, 1.5% EtOH).

### CGRP activation studies

Neutrophils were purified from C57BL6/N bone marrow using negative selection (MojoSort mouse neutrophil purification kit, BioLegend, San Diego, CA, USA) according to the manufacturer’s instructions [67]. 1x10^6^ PMNs were incubated with 100nM or 500nM of CGRP (cat. 1161, R&D Systems, USA), 100nM and 500nM Substance P (cat. 33507-63-1, Millipore Sigma, Darmstadt, Germany) for 6h at 37C. Cells were stimulated with *P*. *aeruginosa* 6294 at MOI of 0.01 for 30 min. Samples were analyzed by flow cytometry.

### CGRP inhibition studies

Mice were injected with CGRP receptor antagonist BIBN4096 (cat. 4096, Tocris, Bristol, UK) intraperitoneally (30 mg/kg) one hour after the infectious challenge [19]. The reagent was prepared on the day of the challenge per manufacturer’s instructions. Control mice were injected with the vehicle (20% DMSO, 1.5% Tween-80 in PBS).

RETRACTED

### Immunohistochemistry of whole mounts and ocular sections

Harvested corneas were fixed for 30 mins in 4% paraformaldehyde (cat.30525-89-4, Alfa Aesar, Ward Hill, MI, USA), washed in PBS, and permeabilized in 1%TritonX100/PBS for 45 min at RT, blocked in 2%BSA, 10% goat serum, 0.1% Triton-x100, PBS, Fc block for 1h, RT. Corneas were then stained with rabbit anti-CGRP (cat. C8198, Sigma, St. Louis, MO, USA) or rabbit anti-beta III tubulin (Tuj1) (ab18207, Abcam, Cambridge, UK) overnight at 4°C, washed, then incubated with goat anti-rabbit IgG-Alexa 568 (Invitrogen, Cambridge, UK) at 4°C overnight. Corneas were subsequently washed, flattened onto slides under a light microscope, and mounted using Prolong anti-fade with DAPI (ThermoFisher, Waltham, MA USA) [6]. The specificity of staining was validated by control staining using non-immune rabbit IgG (cat. 011-000-003, Jackson ImmunoResearch Labs, West Grove, PA, USA). Images were taken on a Zeiss LSM710 confocal microscope with a 40x objective. Z-stacks were acquired from central and peripheral corneas with a comparable thickness of 45 μm across different conditions such as non-infected corneas, shams, infected corneas. Quantification of the neuronal density was done using custom-generated algorithms in Fiji to quantify stained areas of the image on collapsed z-stacks of the corneas. Measurements of neuronal density were in micron per pixel, as previously published [68]. Beta-tubulin III was used as a general neuronal marker.

Ocular tissues including the lids were snap-frozen in liquid nitrogen and, subsequently cryo-sectioned and stained for rat anti-Ly6G-Alexa Fluor-Alexa 594 (Clone 1.8, BioLegend, San Diego, CA, USA), rat anti-CD3-Alexa 594 (clone 17A2, BioLegend, San Diego, CA, USA), rat anti-MHCII-Alexa 594 (clone M5.114. 15.2, BioLegend, San Diego, CA, USA). The individual Ly6G-positive cells, CD3-positive, MHCII-positive cells were counted per section per area. At least 3 consecutive sections per animal were analyzed. Staining controls included isotype stains as per flow cytometry description.

### Capsaicin eye wipe test

The capsaicin eye wipe test was performed three weeks after the RTX treatment. Animals were acclimated to the behavioral testing environment three days before commencing the behavioral test that was performed within the same room as their cage to reduce stress. Mice were gently restrained, 10 μl of 3 mM of a capsaicin solution (Sigma Aldrich, St. Louis, MO, USA) was applied to the left cornea of the mouse. Mice were video recorded during each session immediately after capsaicin application [69]. Observers unaware of treatment counted the number of wipes (via the ipsilateral forepaw) within a minute after application of the solution. Normal facial grooming behavior was not included.

RETRACTED

### Corneal sensitivity

Blink thresholds were measured using a Luneau Cochet-Bonnet esthesiometer (cat. WO-7760; Western Ophthalmics, Lynnwood, WA, USA). The nylon filament, which ranged in length from 0.5 cm to 6.0 cm, was applied to the surface of the central cornea until mice blinked demonstrating a positive response. An absence of a blink reflex resulted in a negative response score of zero [70].

### Trigeminal ganglia primary neurons cultures

Mice were euthanized by CO_2_ inhalation followed by cervical dislocation, and perfused with cold HBSS^-/-^. The trigeminal ganglia (TG) were dissected from the base of the skull and enzymatically dissociated by incubation at 37°C in HEPES-buffered saline (Sigma-Aldrich) containing Collagenase A (cat. 10 103 578 001, Sigma-Roche, St. Louis, MO, USA) (1 mg/kg), and Dispase II (cat. 17105041, Thermo-Fisher, Waltham, MA, USA) (2.4 U/mL) for 30 min at 37°C [59]. Cells were transferred to a tube of DMEM, 10% FBS (Thermo Fisher, Waltham, MA, USA), containing DNase I (cat. 79254, QIAGEN Inc, Germantown, MD, USA) (150U/mL) and dissociated with syringe needles of decreasing gauge to create single cell suspensions. Single-cell suspensions were carefully pipetted over a 15% gradient of Bovine Serum Albumin (BSA) (cat. 12–657 Millipore/Sigma, St. Louis, MO, USA) [27]. The top layers containing the cellular debris were removed and the pellet was washed, re-pelleted, and resuspended in Neuro-Basal-A Medium (NBM) (Thermo Fisher, Waltham, MA, USA). Primary cells were then plated onto laminin (20 μg/mL, Thermo Fisher, Waltham, MA, USA) coated cell culture plates (Westnet, Canton, MA, USA) in NBM with B-27 supplement (2%, Thermo Fisher, Waltham, MA, USA), L-glutamine (2 mM, Thermo Fisher, Waltham, MA, USA), NGF (50 ng/mL, Thermo Fisher, Waltham, MA, USA). For calcium imaging, 3,000 neurons were plated in 35-mm cell culture dishes and used within 24 hours after plating. For *in vitro* CGRP assays, 5,000 neurons were plated per well in a 96 well plate and were cultured for one week. Half of the medium was replaced with a fresh medium every 48 hours.

### Calcium imaging of primary TG neurons

TG neurons were used for calcium imaging within 24 hours after plating. Cultured TG neurons were loaded with 5 uM Fura-2 AM (LifeTechnologies, Carlsbad, CA, USA) in NBM for 30 minutes at 37°C in the dark, gently washed three times, and covered with Krebs-Ringer solution (Boston BioProducts, Ashland, MA, USA) (KR: 120mM NaCl, 5.5 mM HEPES, 1mM D-glucose, pH 7.2) at room temperature, imaged using an Eclipse Ti-S/L100 inverted microscope equipped with a Zyla sCMOS camera (Andor). Cells were illuminated by an ultraviolet light source (Lambda XL lamp, Sutter Instrument), 340 nm and 380 nm excitation alternated by LEPMAC5000 filter wheel (Spectra services). 340/380 ratiometric images were processed, background corrected and analyzed with NIS-elements Advanced Research software (Nikon). To measure calcium flux in response to the bacterial application, bacterial strains, including 6294 (clinical isolate), PAK, PAK Δ*pilA*, PAK Δ*fliC*, and PAK Δ*exsA* were grown overnight in TSA 5% Sheep Blood plates (Fisher Scientific, Hampton, NH, USA) at 37°C, re-suspended in Krebs-Ringer solution to an OD of 0.45 at 650 nm. Measurements were standardized by time of application of Krebs-Ringer, bacterial inoculum, mustard oil, capsaicin, and KCl. NIS-elements software was used to collect and process images and 340/380 ratiometric analysis. The ratios were normalized by a baseline measurement 2 minutes before application of the inoculum. An increase in 340/380 ratio of 25% or more from baseline levels was considered a positive response.

RETRACTED

### *In vitro* CGRP release assay

Trigeminal ganglia neurons were cultured in NBM media with supplements as described above. Neuronal cells were stimulated with an inoculum of *P*. *aeruginosa* 6294 at 5x10^3^ CFU/ml for 30 minutes at 37°C with 5% of CO_2_. The supernatant of each well was aliquoted to a sterile 1.5mL Eppendorf tube, centrifuged at 10,000 rpm for 5 minutes at 4°C, and 50 μL of the supernatant was taken and quantified for CGRP concentration by using a CGRP Enzyme-Linked Immunosorbent kit per manufacturer’s instructions (cat. 589001, Cayman Chemical, Ann Arbor, MI, USA).

### Statistical analysis

Statistical significance of corneal pathology scores, bacterial burden, and cytokine levels was evaluated using Mann-Whitney U test for non-parametric pair-wise comparisons or Kruskal-Wallis non-parametric ANOVA with Dunn’s correction for multigroup comparisons or individual 2-group comparisons (Prism 8.0). For analysis of the bactericidal activity assays, the unpaired Student’s *t*-test was used. Differences were considered significant if the p-values were <0.05.

## Supporting information

S1 Fig RTX-treated mice show reduced eye wipe response to capsaicin challenge. Three weeks after the RTX challenge, the number of eye wipes were counted upon 3 mM capsaicin application onto corneas of RTX-treated or vehicle-treated mice. The eye wiping behavior was monitored for 60-sec post-challenge by a treatment-blinded investigator. Eight animals per cohort were analyzed. Each data point represents an individual mouse. Data are representative from one experiment out of three independent experiments. Bars represent means; error bars, ±SD; symbols, individual mouse. Student’s *t*-test, p = 0.0125. Data demonstrate that the RTX treatment reduces corneal sensitivity to capsaicin challenge which may be associated with the loss of capsaicin-responsive TRPV1^+^ nociceptors.
(EPS)

S2 Fig No major changes in the frequency of Ly6G+ cells in RTX-treated mice and vehicle-treated mice. **A.** Number of Ly6G^+^ cells counted per anatomical area per section. Cornea, fornix tartalis (Ft), fornix bulbi (Fb), and limbal areas were compared. **B.** Representative images from immunohistochemical analysis for Ly6G^+^ cells in the ocular tissues of non-infected RTX and vehicle-treated mice. Ocular tissues were harvested from non-infected RTX (n = 5) and Vehicle-treated (n = 5) mice, cryo-embedded, sectioned, and stained for Ly6G and nucleus (DAPI). The presence of Ly6G positive cells was quantified in three consecutive sections per eye per animal and the mean values were compared across different treatment groups (RTX, vehicle, naïve (non-treated) mice). Abbreviations: L- lid; Li-limbus; C-cornea; Fb-fornix bulbi; CB-ciliary body; Ft-fornix tartalis. No differences were observed in the number of Ly6G^+^ cells in the Fb, Ft, and central cornea, while the number of Ly6G^+^ cells was mildly reduced in the limbus (One-way ANOVA).
(EPS)

S3 Fig No major changes in CD3+ frequencies in RTX-treated mice and vehicle-treated mice. **A.** Number of CD3^+^ cells counted per anatomical area per section. Cornea, Ft, Fb, and limbal areas were compared. **B.** Representative images from immunohistochemical analysis for CD3^+^ cells in the ocular tissues of non-infected RTX- and vehicle-treated mice. Ocular tissues were harvested from non-infected RTX- (n = 5) and vehicle-treated (n = 5) mice were cryo-embedded, sectioned, and stained for CD3 and nucleus (DAPI). The presence of CD3^+^ positive cells was quantified in three consecutive sections per eye (total of 15 sections per treatment group) and the mean values were compared across the different animals. Abbreviations: L- lid; Li-limbus; C-cornea; Ft-fornix bulbi; CB-ciliary body; Ft-fornix tartalis. No differences were observed in the number of CD3^+^ cells in the Fb, Ft, central cornea, and limbus (One-way ANOVA).
(EPS)

S4 Fig No major changes in CD11c+MHCII+ cell frequencies in RTX-treated mice and vehicle-treated mice. **A.** Number of CD11c^+^MHCII^+^ cells counted per anatomical area per section. Cornea, Ft, Fb, and limbal areas were compared. **B.** Representative images from immunohistochemical analysis for CD11c^+^MHCII^+^ in the ocular tissues of non-infected RTX- and vehicle-treated mice. Ocular tissues were harvested from non-infected RTX (n = 5) and vehicle-treated (n = 5) mice were cryo-embedded, sectioned, and stained for CD11c, MHCII, and nucleus (DAPI). The presence of CD11c^+^MHCII^+^ positive cells was quantified in three consecutive sections per eye (total of 15 sections per treatment group) and the mean values were compared across the different animals. Abbreviations: L- lid; Li-limbus; C-cornea; Ft-fornix bulbi; CB-ciliary body; Ft-fornix tartalis. No differences were observed in the number of CD11c^+^MHCII^+^ cells in the Fb, Ft, central cornea, and limbus (One-way ANOVA).
(EPS)

S5 Fig ICAM-1+ PMNs are tissue-specific. **A.** Flow cytometry analysis of PMNs from bone marrow (BM), blood, and corneas from infected C57BL6/N mice. Panels describe the gating strategy to identify neutrophil subpopulations. PMNs were defined on FSC vs SSC gate, as CD45^+^, live cells that express CD11b and Ly6G. Histograms show levels of ICAM-1 presence. **B.** Quantification of ICAM-1^+^ MFI. Bar graphs show mean values. Data are cumulative of values from at least 5 infected mice per experiment and representative of two independent experiments. One-way ANOVA, p = 0.0001. Data demonstrate that ICAM-1 presence is upregulated in the infected corneas.
(EPS)

S6 Fig Lack of RTX-dependent regulation of innate immunity at 48h post-infectious challenge. **A.** Mice were infected with 5x10^5^ CFU/ml of *P*. *aeruginosa* 6294 and corneas were harvested at 48h post-challenge (N = 7 per group). Bacterial burdens (bar with whiskers) were measured, Student’s *t*-test, ns, not significant. Ocular pathology (Mann-Whitney test), ns, not significant. Data are representative of three experiments. **B.** IL-1β, IL-6, KC, MCP, and NE were measured in combined corneal and conjunctival tissue lysates of *P*. *aeruginosa*–infected mice at 48h post-challenge. Student’s *t*-test, ns, not significant. Data are representative of two independent experiments. Cumulatively data shows that nociceptor depletion did not affect bacterial presence at later stages of infection.
(EPS)

S1 Video Representative z-stacks from vehicle-treated shams. Eyes were scratched and corneas harvested 24h post-treatment. Corneal whole mounts were stained for β-tubulin and nucleus (DAPI). The 3D videos were composed in Fiji. The z-stacks were defined by the DAPI layers and ran for 40μm in depth with a spacing of 1μm. The images rotate with increments of 10^0^.
(AVI)

S2 Video Representative z-stacks from RTX-treated shams. Eyes were scratched and corneas harvested 24h post-treatment. Corneal whole mounts were stained for β-tubulin and nucleus (DAPI). The 3D videos were composed in Fiji. The z-stacks were defined by the DAPI layers and ran for 40μm in depth with a spacing of 1μm. The images rotate with increments of 10^0^.
(AVI)

S3 Video Representative z-stacks from vehicle-treated infected corneas. Eyes were scratched and infected with *P*. *aeruginosa* 6294; corneas were harvested 24h post-treatment. Corneal whole mounts were stained for β-tubulin and nucleus (DAPI). The 3D videos were composed in Fiji. The z-stacks were defined by the DAPI layers and ran for 50μm in depth with a spacing of 1μm. The images rotate with increments of 10^0^.
(AVI)

S4 Video Representative z stacks from RTX-treated infected corneas. Eyes were scratched and infected with *P*. *aeruginosa* 6294; corneas were harvested 24h post-treatment. Corneal whole mounts were stained for β-tubulin and nucleus (DAPI). The 3D videos were composed in Fiji. The z-stacks were defined by the DAPI layers and ran for 50μm in depth with a spacing of 1μm. The images rotate with increments of 10^0^.
(AVI)
